The article "Registered Trials of Artificial Intelligence Conducted on Chronic Liver Disease: A Cross-Sectional Study on ClinicalTrials.gov" was retracted in 2023. Reasons: unreliable results or conclusions; concerns about the data; concerns about the peer review; concerns about the citations.

# Registered Trials of Artificial Intelligence Conducted on Chronic Liver Disease: A Cross-Sectional Study on ClinicalTrials.gov

**DOI:** 10.1155/2022/6847073

**Published:** 2022-09-20

**Authors:** Gezhi Zheng, Lei Shi, Jinfeng Liu, Yingren Zhao, Fenjing Du, Yingli He, Xin Yang, Ning Song, Juan Wen, Heng Gao

**Affiliations:** ^1^Department of Infectious Diseases, The First Affiliated Hospital of Xi'an Jiaotong University, China; ^2^The First Affiliated Hospital of Xi'an Jiaotong University Xi'an Health School, China

## Abstract

**Background:**

Artificial intelligence (AI) has been widely applied in the diagnosis and therapy of chronic liver disease (CLD), but there is currently little insight into the trials registered on ClinicalTrials.gov. Thus, this cross-sectional study was focused on analyzing the progress in the use of AI in CLD.

**Methods:**

Registered trials of AI applied in CLD on ClinicalTrials.gov were searched firstly. All available information was downloaded to Excel (Microsoft Excel, Rong, Rong, China), and duplicates were removed. We extracted the data of the included trials, then analyzed the characteristics of them finally.

**Results:**

Up to the 27th of May 2021, 6835 trials were identified following an initial search, and 20 registered trials were included after screening for inclusion and exclusion criteria. Among those trials, hepatocellular carcinoma (HCC, 40.0%) and nonalcoholic fatty liver disease (NAFLD, 20.0%) were the most widely applied CLDs for AI. Trials started in 2013 until 2021, with 17 trials (85%) registered after 2016. There was a large trend in trial enrolment, with 40% of them including samples more than 500. Five trials (25%) have been completed, but only one of these had available results. The most frequent sponsors and collaborators were both hospitals at 55%, followed by universities at 35% and institutes at 11%, respectively. Of the 20 trials included, 35% (7 trials) were interventional trials and 65% (13 trials) were observational trials. Among 7 interventional trials, most trials were for diagnosis purpose (42.86%, 3 trials); 4 trials (57.14%) were randomized; 3 trials (42.86%) applied behavioral intervention, 1 trial (14.29%) was in device intervention, 2 trials (28.57%) were in diagnostic test, and 1 trial intervention was unknown. Among 13 observational trials, 8 (61.54%) were cohort studies; 6 (46.15%) were prospective studies, 4 (30.77%) were retrospective studies, 2 (15.38%) were cross-sectional studies, and 1 (7.69%) did not involve a temporal perspective.

**Conclusion:**

The study is the first to focus on AI registration trials in CLD, which will aid relevant scholars in understanding the current state of the subject. This study demonstrates that additional research on AI used in the diagnosis and treatment of CLD is required, and timely publication of accessible results from registered trials is essential.

The article "Registered Trials of Artificial Intelligence Conducted on Chronic Liver Disease: A Cross-Sectional Study on ClinicalTrials.gov" was retracted in 2023. Reasons: unreliable results or conclusions; concerns about the data; concerns about the peer review; concerns about the citations.

## 1. Introduction

Chronic liver disease is a collective term for a chronic, progressive disease with diffuse fibrosis caused by one or more causes, with the histological features of the liver tissue as the main body and impairment of liver function as the main pathological change. Chronic liver disease is a common chronic disease in China, with a high morbidity and mortality rate, presenting an increasing trend year by year, which has seriously affected the physical and mental health of the Chinese people. Most of chronic liver diseases are caused by the delay of acute liver disease, the pathogenesis is complex, and clinical symptoms such as flank pain, fatigue, weakness, and digestive system symptoms are common, which brings great harm to people's physical and mental health. If not effectively treated, chronic liver disease will gradually develop from mild to severe and eventually develop into cirrhosis and liver cancer, with a poor prognosis and a great impact on patients' lives. Prevention and treatment of chronic liver disease are therefore essential and urgent. Nowadays, Chinese medicine has rich theoretical and clinical experience in the diagnosis and treatment of chronic liver diseases and has made certain progress. Although there is no clear definition or name for chronic liver disease in Chinese medicine, according to the different characteristics of its clinical manifestations, it is mostly classified as “dysthymia,” “jaundice,” “dropsy,” and “accumulation” in traditional Chinese medicine (TCM). Chinese medicine believes that the deficiency of positive energy is the intrinsic basis for the development of chronic liver disease, while factors such as depression, overwork and excessive desire, and uncontrolled diet are the internal causes and dampness, heat, and epidemic toxins are the external causes, which combine to cause the disease, damaging the liver meridians and injuring the liver channels.

Modern medicine generates wealth of patient data that many clinical practitioners find difficult to manipulate and synthesize into actionable knowledge, and in recent years, artificial intelligence (AI) has become an effective tool in this regard [1]. The term “artificial intelligence” was coined in 1955 and defined as “the science and engineering of making intelligent machines,” which implies “the use of a computer to model intelligent behavior with minimal human intervention” [2]. AI is currently utilized in healthcare in a variety of ways, including machine learning (ML), which gathers patient data to formulate mathematical models and predict outcomes. Neural networks (NN) and deep learning (DL) are subsets of machine learning (ML), a more contemporary use of ML that is particularly useful for vast volumes of complex multidimensional data. Neural language processing (NLP) could automatically extract meaningful information from clinical characteristics for clinical monitoring or other purposes [1]..

The article "Registered Trials of Artificial Intelligence Conducted on Chronic Liver Disease: A Cross-Sectional Study on ClinicalTrials.gov" was retracted in 2023. Reasons: unreliable results or conclusions; concerns about the data; concerns about the peer review; concerns about the citations.

Chronic liver disease (CLD) has multiple etiologies, including viral hepatitis, nonalcoholic fatty liver disease (NAFLD), alcoholic liver disease, autoimmune liver disease, and genetic causes such as hereditary hemochromatosis; moreover, it is essentially a progressive deterioration in liver functions leading to fibrosis and cirrhosis [3], and hepatocellular carcinoma (HCC) is a potentially fatal consequence of CLD. AI in hepatology not only could accomplish early detection and treatment of CLD, thereby delaying and reducing the incidence of cirrhosis and HCC, but also reduces the necessity for intrusive measurements such as biopsy and catheterization to evaluate hepatic venous pressure gradients (HVPG). There are a rising number of published studies; for instance, a research in chronic viral hepatitis conducted by Runmin et al. using basic characteristics such as age, transaminases, albumin, and platelet counts found that ML was superior to FIB-4 in predicting liver fibrosis [4]. As for NAFLD, ML could not be only as a screening tool based on gender, age, BMI, abdominal girth, glucose, lipid profile, and GGT [5] but also as an indicator to distinguish patients with nonalcoholic steatohepatitis (NASH) in patients with NAFLD [6]. Singal et al. followed up 442 patients with cirrhosis and developed a machine learning algorithms (MLAs) for predicting HCC, which showed better performance compared to traditional methods [7]. MLAs are also serving as measurements for the selection of liver transplant (LT) recipients and assessing posttransplant outcomes [8]. The use of image-based AI (HVPG) could also reduce invasive measurements such as biopsies and catheterization to measure the hepatic venous pressure gradient. For example, ultrasound-based MLA is more accurate in detecting steatosis, hepatic fibrosis, and localized liver lesions [9–11]. Several studies have demonstrated the efficiency of support vector machine (SVM) models based on magnetic resonance (MR) images and convolutional neural network (CNN) models based on computed tomography (CT) images in predicting and staging liver fibrosis [12–14]. Other investigators have demonstrated in previous studies that SVM models based on digital pathology images may detect steatosis and assess the degree of liver fibrosis [15, 16]. Liu et al. reported that CNN based on CT or MR could identify clinically significant portal hypertension (CSPH) in patients with cirrhosis accurately [17].

The article "Registered Trials of Artificial Intelligence Conducted on Chronic Liver Disease: A Cross-Sectional Study on ClinicalTrials.gov" was retracted in 2023. Reasons: unreliable results or conclusions; concerns about the data; concerns about the peer review; concerns about the citations.

ClinicalTrials.gov is a database of private and public funded clinical research conducted worldwide [18]; the researches on this website are transparent and traceable, analyzing registered trials on that will provide the progress of one field. A variety of articles have been published on ClinicalTrials.gov to analyze registered trials [19–23]. AI has been widely applied in the diagnosis and treatment of CLD, and the current research is addressing a range of issues and will lead to greater achievement, but few trials registered with ClinicalTrials.gov are currently known to the academic community. Thus, we focused this cross-sectional study on the analysis of the progress of AI applied in CLD.

## 2. Materials and Methods

### 2.1. Data Search

Registered trials on ClinicalTrials.gov were searched according to the following terms: AI, artificial intelligence, computational intelligence, computer reasoning, computer vision system, deep learning, knowledge representation (computer), knowledge acquisition (computer), machine intelligence, machine learning, natural language processing, neural network, algorithms, and neural networks of computer and robotics. All available information was downloaded to Excel (Microsoft Excel, Rong, Rong, China), and duplicates were removed via Excel based on the trials' national clinical trial (NCT) number.

The trial was conducted in accordance with Clinical Practice guidelines established by the International Council for Harmonisation and in compliance with the trial protocol. The protocol was approved by the institutional review boards or independent ethics committees at each site (Approval No. NI-YU20200201). All patients provided written informed consent per Declaration of Helsinki principles. An independent data monitoring committee monitored safety and efficacy data.

### 2.2. Inclusion and Exclusion Criteria

The inclusion criteria were registered trials for AI conducted on the CLD based on the “conditions” in Excel. Two authors (Zhang Xiaoli and BAIMA Yangjin) then independently and meticulously screened each trial to exclude those unrelated of AI.

### 2.3. Data Extraction and Analysis

Data were extracted from the included trials. For interventional studies, the following information was extracted: type of liver disease, study type, registered year, enrollment, participant gender, participant age, status, applications, study results, sponsors and collaborators, locations, primary purpose, interventions, intervention model, allocation, masking, and time perspective.

The article "Registered Trials of Artificial Intelligence Conducted on Chronic Liver Disease: A Cross-Sectional Study on ClinicalTrials.gov" was retracted in 2023. Reasons: unreliable results or conclusions; concerns about the data; concerns about the peer review; concerns about the citations.

For observational studies, the following information was extracted: observational model and time perspective.

As this was a cross-sectional study, the characteristics of the registered trials were analyzed using descriptive analysis.

## 3. Results

### 3.1. Basic Characteristics

As of 27^th^ May 2021, 6835 trials were identified following the initial search. A total of 20 registered trials were included based on inclusion and excluding criteria, as shown in Figure 1. The types of CLDs and methods of application are shown in Table 1, with NAFLD (4 trials, 20.0%) and HCC (8 trials, 40.0%) being the CLDs in which AI was most widely applied; imaging was most commonly used in the application of AI in CLD. The characteristics of the included trials are shown in Table 2. Trials started from 2013 to 2021, and 17 trials (85%) were registered after 2016. Enrollment in trials tended to be large, with 10 (50%) studies including cases ranging from 100 to 500, of which 40% included samples of more than 500. Four trials remained unrecruited, 11 trials were in recruitment, and 5 trials have been completed, but among them, only 1 trial had available results. The most common sponsors and collaborators were both hospitals at 55%, followed by universities at 35% and research institutes at 11%, respectively. Out of the 20 included trials, 35% (7 trials) were interventional and 65% (13 trials) were observational trials; furthermore, we have also analyzed the characteristics of them, respectively.

### 3.2. Interventional Study

The characteristics of the 7 interventional trials are shown in Table 3. Most trials were for diagnosis (42.86%, 3 trials), 1 was for treatment, 1 was for screening, 1 was for health services research, and 1 trial did not clearly describe the primary purpose clearly. Three trials (42.86%) applied behavioral intervention, 1 (14.29%) was in device intervention, 2 (28.57%) were in diagnostic test, and 1 trial intervention was unknown. As for the model of intervention, 5 (71.43%) were allocated in parallel, 2 (28.57%) were allocated in a single group, and there were no sequential assignment, cross-assignment, and factorial assignment. For allocation, 4 (57.14%) were stochastic, 1 (14.29%) was nonrandomized, and 2 (28.58%) were not applicable. For masking, 2 (28.57%) were single, 1 (14.29%) was double, and 4 (57.14%) were open-labeled.

### 3.3. Observational Study

The characteristics of the 13 observational trials are shown in Table 4. Among the 13 observational studies, 8 (61.54%) were cohort studies, 2 (15.38%) were case-control studies, 1 (7.69%) was a case-only study, and 2 (15.38%) did not specify the observational model. Six (46.15%) trials were prospective studies, 4 (30.77%) were retrospective studies, 2 (15.38%) were cross-sectional studies, and 1 (7.69%) did not refer to the time perspective.

The article "Registered Trials of Artificial Intelligence Conducted on Chronic Liver Disease: A Cross-Sectional Study on ClinicalTrials.gov" was retracted in 2023. Reasons: unreliable results or conclusions; concerns about the data; concerns about the peer review; concerns about the citations.

## 4. Discussion

Chronic liver disease is a collective term for slowly developing, long-standing, and persistently damaging diseases of the liver such as viral hepatitis, nonalcoholic fatty liver disease (NAFLD), liver fibrosis, cirrhosis, and liver cancer. The development of chronic liver disease is a complex process influenced by multiple factors. For different etiologies, the current clinical pharmacological treatment mostly adopts symptomatic management, including hepatoprotection, antiviral, immune modulation, and anti-liver fibrosis. Due to long-term chronic liver inflammatory damage, excessive repair of liver tissue causes the loss of structure and function of liver lobules, forming liver fibrosis, and the continued progression of liver fibrosis leads to the formation of cirrhosis, on top of which the risk of liver cancer increases year by year. Chronic liver disease belongs to the Chinese medicine categories of “dysesthesia,” “accumulation of evidence,” “jaundice,” and “dropsy,” which are mostly caused by deficiency of vital energy, internal stasis of blood, and loss of nourishment in the liver meridian.

AI has been extremely helpful in the assessment of CLDs, with a large number of published studies applying AI to liver disease over the last decade [1, 3–5, 7–17, 24]. To our surprise, only 20 trials for the usage of AI in CLD have been registered on ClinicalTrials.gov. One explanation is that most studies were not registered on ClinicalTrials.gov at the start of the study, as evidenced by the fact that they were published without the NCT number [4, 5, 7–16, 24].. Another reason might be that some of the registered trials on ClinicalTrials.gov published under other title. For example, Liu et al. published a study that developed a CT- or MR-based deep convolutional neural network (CNN) model to identify patients with clinically significant portal hypertension (CSPH) (NCT 03138915 and NCT 03766880) [17]; nevertheless, the results searched on the ClinicalTrials.gov based on the two NCT numbers are not relevant to AI [25, 26].

Among the 20 registered trials, NAFLD (4 trials, 20.0%) and HCC (8 trials, 40.0%) were the CLDs in which AI was most widely applied, with imaging being the most commonly used in the application of AI in CLDs. There were no trials for children only. On the one hand, NAFLD and HCC occur infrequently in children, and on the other hand, studies in children are very challenging given their ethical, scientific, and practical considerations [19, 27]. The majority of trials (85%) were registered after 2017, which coincide with the fourth industrial revolution, that is, AI combined with big data to guide medical information [28]. Our study showed that most trials incorporate large samples (100-500 samples), which may contribute to reduce statistical differences [19, 29].

The article "Registered Trials of Artificial Intelligence Conducted on Chronic Liver Disease: A Cross-Sectional Study on ClinicalTrials.gov" was retracted in 2023. Reasons: unreliable results or conclusions; concerns about the data; concerns about the peer review; concerns about the citations.

In our study, 25% of the researches were completed, but only 5% of the detailed results were available on the ClinicalTrials.gov. The results were similar to the conclusion of Liu et al. [19] and Chen et al. [22], which implies a lack of transparency in these trials. This is probably due to the fact that most researchers would not like to upload negative results, and many studies also reported the phenomenon that negative results do not have chance to be published [30–32]. Ioannidis et al. described the phenomenon as a publication lag, which may significantly reduce the value of evidence and generate bias, as positive results may one-sidedly capture our information systems for a period of time before negative results are published [33]. We discovered that the majority of studies were observational trials (65.0%), although observational studies would cause a series of bias and thus to false results [34], but it was reasonable since it was still at the early stage of application of AI in diagnosis and treatment of CLD, and researches still need build lots of AI models to conduct prospective studies in the future.

Due to the constraints, our study is unlikely to capture the entire extent of this field. For starters, the majority of the trials we looked into did not provide results. Secondly, our search yielded too few trials. On the one hand, despite the fact that ClinicalTrials.gov is the most widely utilized registry site [35],, there are also others, such as the National Institutes of Health (NIH) and Chinese Clinical Trial Registry (ChiCTR), where not all trials are registered on ClinicalTrials.gov. On the other hand, not all researchers registered their trial prior to the study.

The following are the main issues that remain for the extension of AI technology to clinical practice: (1) there is a lack of high-quality training and validation datasets for model development and validation, and there is a need to establish high-quality and accessible research cohorts of patients with chronic liver disease. (2) Most of the models and algorithms developed for liver disease lack long-term evaluation in clinical practice and direct comparison with traditional diagnostic methods, and their performance in the real world has yet to be proven. (3) The technical barriers between algorithm developers and clinicians have yet to be breached, and the interpretability and transparency of AI output conclusions have yet to be improved. (4) In terms of medical ethics, we should consider who should bear the consequences if mistakes are made during the application of AI and what should be done to ensure the maximum benefit for patients. These issues need to be further regulated.

The article "Registered Trials of Artificial Intelligence Conducted on Chronic Liver Disease: A Cross-Sectional Study on ClinicalTrials.gov" was retracted in 2023. Reasons: unreliable results or conclusions; concerns about the data; concerns about the peer review; concerns about the citations.

AI is playing an increasingly important role in the field of chronic liver disease due to its own continuous technological advances and the inherent complexity of the biomedical problem itself, by helping in the diagnostic classification of liver disease, predicting the risk of fibrosis in patients with chronic liver disease, objectively assessing liver imaging, and further refining the histological assessment of the liver. In the future, AI technology will be used to develop more accurate models to predict and monitor liver disease progression and potential complications and to improve the lack of healthcare resources in remote or developing areas. In addition, AI can be applied to drug development, processing microarray data and detecting tumour microenvironment to help liver tumour patients achieve more precise and individualised treatment.

## 5. Conclusion

In summary, this study is the first study to investigate AI-registered trials conducted on CLD, which would help relevant scholars to understand the current situation of this field. Our study demonstrated that more researches are required to focus on AI applied in the diagnosis and treatment of CLD, and it is essential to report available results from registered trials in a timely manner.

## Figures and Tables

**Figure 1:** A total of 20 trials were included.

**Table 1:** Overview of clinical trials in diagnosis.

Characteristics	Number	Percentage (%)
Liver diseases		
Hepatic B/C with/without liver failure or liver fibroses	3	15.00
NAFLD/alcoholic fatty liver with/without liver fibroses	4	20.00
Liver cirrhosis	1	5.00
Liver cancer/HCC	8	40.00
Polycystic liver disease	1	5.00
Liver metastases	1	5.00
Focal liver lesions	2	10.00
Application method		
Imaging	9	45.00
Pathology/biopsy	2	10.00
Biomarker/lab test	4	20.00
Imaging and biomarker/lab test	1	5.00
Other	4	20.00

**Table 2:** The characteristics of the 20 trials on ClinicalTrials.gov.

Characteristics	Number	Percentage (%)
Study type		
Interventional	7	35.00
Observational	13	65.00
Registered year		
2004-2010	0	0
2011-2016	3	15.00
2017-2021	17	85.00
Enrollment		
0-99	2	10.00
100-500	10	50.00
>500	8	40.00
Gender		
Female only	1	5.00
Both	19	95.00
Age		
<18	0	0
≥18	17	85.00
All	3	15.00
Status		
Not recruiting	4	20.00
Recruiting	11	55.00
Completed	5	25.00
Study results		
Has results	1	5.00
No results available	19	95.00
Sponsor		
University	7	35.00
Hospital	11	55.00
Company/industry	1	5.00
Institute	1	5.00
Other	0	0
Collaborators		
University	2	10.00
Hospital	11	55.00
Company/industry	1	5.00
Institute	3	15.00
Other	3	15.00
Location		
America	6	30.00
Europe	7	35.00
Asia	7	35.00

The article "Registered Trials of Artificial Intelligence Conducted on Chronic Liver Disease: A Cross-Sectional Study on ClinicalTrials.gov" was retracted in 2023. Reasons: unreliable results or conclusions; concerns about the data; concerns about the peer review; concerns about the citations.

**Table 3:** Designs of 7 interventional trials registered in ClinicalTrial.gov.

Characteristics	Number	Percentage (%)
Primary purpose		
Diagnosis	3	42.86
Treatment	1	14.29
Screening	1	14.29
Health services research	1	14.29
Other	1	14.29
Intervention		
Behavioral	3	42.86
Device	1	14.29
Diagnostic test	2	28.57
Other	1	14.29
Intervention model		
Parallel assignment	5	71.43
Single group assignment	2	28.57
Sequential assignment	0	0
Crossover assignment	0	0
Factorial assignment	0	0
Allocation		
Randomized	4	57.14
Nonrandomized	1	14.29
N/A	2	28.57
Masking		
Single	2	28.57
Double	1	14.29
None (open-label)	4	57.14
Registered year		
2004-2010	0	0
2011-2016	1	14.29
2017-2021	6	85.71
Enrollment		
0-99	1	14.29
100-500	6	85.71
>500	0	0
Gender		
Female only	1	14.29
Both	6	85.71
Age		
<18	0	0
≥18	7	100.00
All	0	0
Status		
Not recruiting	1	14.29
Recruiting	3	42.86
Completed	3	42.86
Study results		
Has results	1	14.29
No results available	6	85.71
Sponsor		
University	4	57.14
Hospital	2	28.57
Company/industry	1	14.29
Institute	0	0
Other	0	0
Collaborators		
University	1	14.29
Hospital	3	42.86
Company/industry	1	14.29
Institute	2	28.57
Other	0	0
Location		
America	3	42.86
Europe	1	14.29
Asia	3	42.86

**Table 4:** Designs of 13 observational trials registered in ClinicalTrial.gov.

Characteristics	Number	Percentage (%)
Observational model		
Case-only	1	7.69
Case-control	2	15.38
Case-crossover	0	0
Cohort	8	61.54
Other	2	15.38
Time perspective		
Prospective	6	46.15
Retrospective	4	30.77
Cross-sectional	2	15.38
Other	1	7.69
Registered year		
2004-2010	0	0
2011-2016	2	15.38
2017-2021	11	84.62
Enrollment		
0-99	1	7.69
100-500	4	30.77
>500	8	61.54
Gender		
Female only	0	0
Both	13	100.00
Age		
<18	0	0
≥18	10	76.92
All	3	23.08
Status		
Not recruiting	3	23.08
Recruiting	8	61.54
Completed	2	15.38
Study results		
Has results	0	0
No results available	13	100.00
Sponsor		
University	3	23.08
Hospital	9	69.23
Company/industry	0	0
Institute	1	7.69
Other	0	0
Collaborators		
University	1	7.69
Hospital	8	61.54
Company/industry	0	0
Institute	1	7.69
Other	3	23.08
Location		
America	3	23.08
Europe	6	46.15
Asia	4	30.77

## Data Availability

All data generated or analyzed during this study are included in this published article.

## References

[1] Ahn J. C., Connell A., Simonetto D. A., Hughes C., Shah V. H. (2021). Application of artificial intelligence for the diagnosis and treatment of liver diseases. *Hepatology*.

The article "Registered Trials of Artificial Intelligence Conducted on Chronic Liver Disease: A Cross-Sectional Study on ClinicalTrials.gov" was retracted in 2023. Reasons: unreliable results or conclusions; concerns about the data; concerns about the peer review; concerns about the citations.

[2] Hamet P., Tremblay J. (2017). Artificial intelligence in medicine. *Metabolism*.

[3] Sharma A., Nagalli S. (2021). Chronic Liver Disease. *StatPearls*.

[4] Wei R., Wang J., Wang X. (2018). Clinical prediction of HBV and HCV related hepatic fibrosis using machine learning. *eBioMedicine*.

[5] Wu C.-C., Yeh W.-C., Hsu W.-D. (2019). Prediction of fatty liver disease using machine learning algorithms. *Computer Methods and Programs in Biomedicine*.

[6] Garcia-Carretero R., Vigil-Medina L., Barquero-Perez O., Ramos-Lopez J. (2019). Relevant features in nonalcoholic steatohepatitis determined using machine learning for feature selection. *Metabolic Syndrome and Related Disorders*.

[7] Singal A. G., Mukherjee A., Elmunzer B. J. (2013). Machine learning algorithms outperform conventional regression models in predicting development of hepatocellular carcinoma. *The American Journal of Gastroenterology*.

[8] Briceño J., Cruz-Ramírez M., Prieto M. (2014). Use of artificial intelligence as an innovative donor-recipient matching model for liver transplantation: results from a multicenter Spanish study. *Journal of Hepatology*.

[9] Kuppili V., Biswas M., Sreekumar A. (2017). Extreme learning machine framework for risk stratification of fatty liver disease using ultrasound tissue characterization. *Journal of Medical Systems*.

[10] Li W., Huang Y., Zhuang B.-W. (2019). Multiparametric ultrasomics of significant liver fibrosis: a machine learning-based analysis. *European Radiology*.

[11] Schmauch B., Herent P., Jehanno P. (2019). Diagnosis of focal liver lesions from ultrasound using deep learning. *Diagnostic and Interventional Imaging*.

[12] He L., Li H., Dudley J. A. (2019). Machine learning prediction of liver stiffness using clinical and T2-weighted MRI radiomic data. *AJR. American Journal of Roentgenology*.

[13] Ahmed Y., Hussein R. S., Basha T. A. (2020). Detecting liver fibrosis using a machine learning-based approach to the quantification of the heart-induced deformation in tagged MR images. *NMR in Biomedicine*.

[14] Choi K. J., Jang J. K., Lee S. S. (2018). Development and validation of a deep learning system for staging liver fibrosis by using contrast agent-enhanced CT images in the liver. *Radiology*.

[15] Vanderbeck S., Bockhorst J., Komorowski R., Kleiner D. E., Gawrieh S. (2014). Automatic classification of white regions in liver biopsies by supervised machine learning. *Human Pathology*.

[16] Wang T.-H., Chen T.-C., Teng X., Liang K.-H., Yeh C.-T. (2015). Automated biphasic morphological assessment of hepatitis B-related liver fibrosis using second harmonic generation microscopy. *Scientific Reports*.

The article "Registered Trials of Artificial Intelligence Conducted on Chronic Liver Disease: A Cross-Sectional Study on ClinicalTrials.gov" was retracted in 2023. Reasons: unreliable results or conclusions; concerns about the data; concerns about the peer review; concerns about the citations.

[17] Liu Y., Ning Z., Örmeci N. (2020). Deep convolutional neural network-aided detection of portal hypertension in patients with cirrhosis. *Clinical Gastroenterology and Hepatology*.

[18] Home - ClinicalTrials.gov. https://clinicaltrials.gov/.

[19] Liu G., Li N., Chen L., Yang Y., Zhang Y. (2021). Registered trials on artificial intelligence conducted in emergency department and intensive care unit: a cross-sectional study on ClinicalTrials.gov. *Frontiers in medicine*.

[20] Dong J., Geng Y., Lu D. (2020). Clinical trials for artificial intelligence in cancer diagnosis: a cross-sectional study of registered trials in *ClinicalTrials.gov*. *Oncologia*.

[21] Chen J., Huang J., Li J. V., Lv Y., He Y., Zheng Q. (2017). The characteristics of TCM clinical trials: a systematic review of ClinicalTrials.gov. *Evidence-based Complementary and Alternative Medicine*.

[22] Chen L., Su Y., Quan L., Zhang Y., Du L. (2018). Clinical trials focusing on drug control and prevention of ventilator-associated pneumonia: a comprehensive analysis of trials registered on ClinicalTrials.gov. *Frontiers in Pharmacology*.

[23] Chen L., Wang M., Yang Y., Shen J., Zhang Y. (2020). Registered interventional clinical trials for old populations with infectious diseases on ClinicalTrials.Gov: a cross-sectional study. *Frontiers in Pharmacology*.

[24] Chang E. K., Yu C. Y., Clarke R. (2016). Defining a patient population with cirrhosis. *Journal of Clinical Gastroenterology*.

[25] Qi X. (2019). MR-based models for noninvasive detection of clinically significant portal hypertension in cirrhosis (CHESS1802). clinicaltrials.gov. https://clinicaltrials.gov/ct2/show/study/NCT03766880.

[26] Qi X. (2019). Development and validation of a radiomics signature for clinically significant portal hypertension in cirrhosis (CHESS1701): a prospective multicenter study. clinicaltrials.gov. https://clinicaltrials.gov/ct2/show/NCT03138915.

[27] Califf R. M., Zarin D. A., Kramer J. M., Sherman R. E., Aberle L. H., Tasneem A. (2012). Characteristics of clinical trials registered in ClinicalTrials.gov, 2007-2010. *JAMA*.

[28] Jha S., Topol E. J. (2016). Adapting to artificial intelligence. *JAMA*.

[29] Inrig J. K., Califf R. M., Tasneem A. (2014). The landscape of clinical trials in nephrology: a systematic review of clinicaltrials.gov. *American Journal of Kidney Diseases*.

[30] Easterbrook P. J., Berlin J. A., Gopalan R., Matthews D. R. (1991). Publication bias in clinical research. *Lancet*.

[31] Dickersin K. (1990). The existence of publication bias and risk factors for its occurrence. *JAMA*.

[32] Dickersin K., Min Y. I., Meinert C. L. (1992). Factors influencing publication of research results. *JAMA*.

The article "Registered Trials of Artificial Intelligence Conducted on Chronic Liver Disease: A Cross-Sectional Study on ClinicalTrials.gov" was retracted in 2023. Reasons: unreliable results or conclusions; concerns about the data; concerns about the peer review; concerns about the citations.

[33] Ioannidis J. P. (1998). Effect of the statistical significance of results on the time to completion and publication of randomized efficacy trials. *JAMA*.

[34] Hammer G. P., du Prel J.-B., Blettner M. (2009). Avoiding bias in observational studies: part 8 in a series of articles on evaluation of scientific publications. *Deutsches Ärzteblatt International*.

[35] Zarin D. A., Ide N. C., Tse T., Harlan W. R., West J. C., Lindberg D. A. B. (2007). Issues in the registration of clinical trials. *JAMA*.

